# Effects of Cisplatin Combined with Metformin on Proliferation and Apoptosis of Nasopharyngeal Carcinoma Cells

**DOI:** 10.1155/2022/2056247

**Published:** 2022-04-05

**Authors:** Ling Shi, Yaoguo Mei, Xunhuang Duan, Bo Wang

**Affiliations:** ^1^Department of Oncology, First People's Hospital of Jiujiang City, Jiujiang, 332000 Jiangxi Province, China; ^2^Department of Oncology, Jiujiang Hospital of Traditional Chinese Medicine, Jiujiang, 332000 Jiangxi Province, China

## Abstract

**Background:**

Nasopharyngeal carcinoma (NPC) is an invasive squamous cell carcinoma located in the nasopharynx. NPC has a high recurrence risk after initial treatment due to its high metastatic and immune escape potential. One study has found that metformin can improve cancer outcomes and reduce cancer incidence.

**Objective:**

With antitumor activity, metformin can have low toxicity when used in combination with some common chemotherapy drugs. This study was designed to explore the effects of cisplatin combined with metformin on the proliferation and apoptosis of nasopharyngeal carcinoma (NPC) cells.

**Methods:**

An appropriate cisplatin concentration was selected for NPC cells, and the cells were treated with metformin at a gradient concentration, and then, some of them were treated with cisplatin. Subsequently, the biological effects (activity, migration, invasion, and apoptosis) of metformin alone and metformin combined with cisplatin on NPC cells were evaluated.

**Results:**

Metformin alone inhibited cell activity, migration, and invasion and promoted cell apoptosis in a concentration-dependent and time-dependent manner, while compared with cisplatin alone, cisplatin combined with metformin had stronger inhibition on cell activity, migration, and invasion and stronger induction to cell apoptosis, and a higher concentration of them demonstrated stronger effects.

**Conclusion:**

Cisplatin combined with metformin can strongly inhibit the activity of NPC cells and promote their apoptosis.

## 1. Introduction

Nasopharyngeal carcinoma (NPC) is an invasive squamous cell carcinoma located in the nasopharynx [1]. As a rare malignant tumor [2], it is treated differently from other head and neck carcinomas [3]. NPC is difficult to detect and diagnose early due to its insidious lesion in the nasopharynx cavity and insignificant early symptoms [4], and it has a high recurrence risk after initial treatment due to its high metastatic and immune escape potential [5]. At present, NPC is mainly treated by radiotherapy and chemotherapy.

Cisplatin, a common chemotherapy drug, has been widely applied to treat various cancers [6]. It mediates its antitumor effect through many different cytotoxic mechanisms, and in addition to resulting in DNA damage, it also causes dysfunction of cytoplasm, activates apoptosis pathways, and gives rise to cell damage via oxidative stress and inflammation [7]. Cisplatin is effective in treating tumors, but it has strong toxic and side effects. Metformin is a widely used drug that can provide obvious benefits in glucose metabolism and diabetes mellitus-related complications [8]. One study has found that metformin can improve cancer outcomes and reduce cancer incidence. It not only can reduce plasma glucose levels in several mechanisms but also is characterized by being able to favorably regulate serum lipids, reduce endothelial inflammatory cell adhesion, and exert anti-inflammatory, antiapoptosis, and antioxidant properties [9]. One study has pointed out that the use of metformin is associated with a relatively low incidence of cancer in diabetic patients and is considered useful for cancer therapy in nondiabetic patients [10], and one other study has revealed that in breast cancer models, metformin can delay the onset of breast cancer and prolong the average life span of patients with breast cancer by 8% [11], which both indicate that metformin has important anticancer properties. However, a considerable number of clinical trials of single-dose metformin failed to demonstrate a convincing efficiency of metformin. Therefore, recent studies tend to combine metformin with a commonly used chemotherapy drug in clinical practice to reduce the toxicity of metformin and tumor resistance to it [12]. In addition, in order to minimize the side effects of cisplatin and resistance to it clinically, combination therapy has also been applied and it has been verified to be more effective in the treatment of cancers [13]. This study was designed to explore the biological effects of cisplatin combined with metformin on NPC cells.

## 2. Methods

### 2.1. Materials

NPC cell lines (CNE1) (Beinuo Biotechnology Co., Ltd., Shanghai, China), metformin hydrochloride (State Food and Drug Administration (SFDA) approval number: H20023370, Sino-American Shanghai Squibb Pharmaceutical Co., Ltd., Shanghai, China), cisplatin injection (SFDA approval number: H53021741, Yunnan Phytopharmaceutical Co., Ltd., Yunnan, China), Dulbecco's modified Eagle medium (DMEM) (Chuan Qiu Biotechnology Co., Ltd., Shanghai, China), apoptosis kit (Chreagen Biotechnology Co., Ltd., Beijing, China), microplate reader (Yanhui Biotechnology Co., Ltd., Shanghai, China), 10% fetal bovine serum (FBS; AMEKO Biotechnology Co., Ltd., Shanghai, China), cell counting kit-8 (CCK8) (Yubo Biological Technology Co., Ltd., Shanghai, China), BD flow cytometer (Derica Biotechnology Co., Ltd., Beijing, China), Transwell chamber (Ziqi Biotechnology Co., Ltd., Shanghai, China), trypsin (Yuanye Biotechnology Co., Ltd., Shanghai, China), and penicillin streptomycin (Yuanye Biotechnology Co., Ltd., Shanghai, China) were used.

### 2.2. Methods

#### 2.2.1. Cell Culturing

Serial subcultivation was carried out in high-sugar DMEM containing 10% FBS+1% penicillin/streptomycin solution. Cells were cultured in a culture flask first and then digested with trypsin when they were in a good growth state, counted, and seeded to a plate for culture for subsequent analysis. In this assay, the action time of drugs on cells was 24 h.

#### 2.2.2. Cell Activity Determination by CCK8

Cell activity was determined using CCK8. CNE1 cells were cultured in a 96-well plate until they reached 80% confluency, and then, they were treated with 0.5-10 mg cisplatin. After 24 h and 48 h of treatment, the cell activity was determined. It came out that when the concentration of cisplatin was below 2 mg/L, the cell activity was basically above 90%, so the effect of cisplatin on cell activity was small at this time. However, when the concentration of cisplatin was above 2 mg/L, the cell activity was inversely proportional to the concentration of cisplatin. Therefore, in this assay, we select 2 mg/L cisplatin for subsequent experiments (Figure 1). Afterwards, CNE1 cells were treated with metformin (0.01, 0.5, 1, and 5 mmol/L) or cisplatin (2 mg/L). Each well was added with 10 mL CCK8 solution diluted with 100 mL FBS-free DMEM at 1 : 10 at 24, 48, and 72 h after culturing according to the manufacturer's guidelines, and then, the cells were cultured under the same conditions for another 1 hour. The optical density (OD) of cells at 450 nm was measured using the microplate reader. The average OD of shown groups was used to calculate the percentage of cell activity.

#### 2.2.3. Detection of Cell Migration and Invasion

The cell suspension was transferred to the upper compartment with serum-free medium at 5 × 10^4^ cells/well, and the lower compartment was added with a medium containing 10% FBS as a chemical attractant. Cells that did not migrate after 24 hours of culture were removed from the upper surface of the filter by swabbing, and then, the membrane was immobilized with 4% formaldehyde for 15 min at indoor temperature and dyed with 0.5% crystal violet for 15 min. For the determination of cell invasion, based on the above steps, 8% Matrigel was applied.

#### 2.2.4. Cell Apoptosis Assay

The number of apoptotic cells was determined using flow cytometry. After 72 hours of treatment with metformin (0.5, 1, and 5 mmol/L) and cisplatin (2 mg/L), cells were digested with trypsin and harvested and then washed with PBS twice and suspended in trypsin-ethylenediaminetetraacetic acid (EDTA) solution (containing 0.25% trypsin and 0.02% EDTA) binding buffer (1 × 10^6^ cells/mL). The cells were added with Annexin V and PI and then incubated in the dark at room temperature for 15 min. Finally, the cells were analyzed by a flow cytometer.

### 2.3. Statistical Analysis

Differences were verified by SPSS 21.0 (SPSS, Inc., Chicago, IL, USA), and measurement data were analyzed using the *t*-test and expressed as the mean ± standard deviation (*x* ± sd). Comparison within groups at different time points was carried out using the repeated measures analysis of variance. *p* < 0.05 indicates a significant difference.

## 3. Results

### 3.1. Metformin Combined with Cisplatin Inhibited Activity of CNE1 Cells

We analyzed the effects of metformin and cisplatin on the activity of CNE1 cells, finding that metformin alone significantly inhibited the activity of CNE1 cells in a time- and concentration-dependent manner (Figure 2), and compared with cisplatin alone, the activity of CNE1 cells decreased with the increase of the concentration of metformin combined with cisplatin (Figure 3), which indicated that metformin combined with cisplatin could effectively inhibit the activity of NPC cells. The activity of CNE1 cells treated with metformin alone decreased significantly with the increase of time and also decreased with the increase of metformin concentration. Compared with cisplatin alone, the activity of CNE1 cells decreased with the increase of the concentration of metformin combined with cisplatin.

### 3.2. Metformin Combined with Cisplatin Inhibited Migration of CNE1 Cells

Determination of the effect of metformin and cisplatin on the migration of CNE1 cells revealed that metformin alone exerted a strong inhibition on the migration of CNE1 cells, and the inhibition intensity increased with the increase of concentration (Figure 4), and compared with cisplatin alone, metformin combined with cisplatin inhibited cell migration in a concentration-dependent manner (Figure 5), which indicated that metformin combined with cisplatin could strongly inhibit the migration of NPC cells. Compared with the control group, the migration of cells treated with metformin alone was inhibited, and the inhibition intensity increased with the increase of concentration. Compared with the control group, cisplatin significantly inhibited cell migration, and compared with cisplatin alone, cisplatin combined with metformin inhibited cell migration more significantly.

### 3.3. Metformin Combined with Cisplatin Inhibited Invasion of CNE1 Cells

Determination of the effect of metformin and cisplatin on the invasion of CNE1 cells revealed that metformin alone exerted a strong inhibition on the invasion of CNE1 cells, and the inhibition intensity increased with the increase of concentration (Figure 6), and compared with cisplatin alone, metformin combined with cisplatin inhibited cell invasion in a concentration-dependent manner (Figure 7), which indicated that metformin combined with cisplatin could strongly inhibit the invasion of NPC cells. Compared with the control group, the invasion of cells treated with metformin alone was inhibited, and the inhibition intensity increased with the increase of concentration. Compared with the control group, cisplatin significantly inhibited cell invasion, and compared with cisplatin alone, cisplatin combined with metformin inhibited cell invasion more significantly.

### 3.4. Metformin Combined with Cisplatin Induced Apoptosis of CNE1 Cells

Determination of the effect of metformin and cisplatin on the apoptosis of CNE1 cells revealed that metformin alone induced the apoptosis of CNE1 cells, and the apoptosis rate increased with the increase of concentration (Figure 8), and compared with cisplatin alone, metformin combined with cisplatin induced cell apoptosis in a concentration-dependent manner (Figure 9), which indicated that metformin combined with cisplatin could induce the apoptosis of NPC cells. Compared with the control group, the apoptosis of cells treated with metformin alone increased, and the cell apoptosis increased with the increase of metformin concentration. Compared with the control group, cisplatin significantly promoted cell apoptosis, and compared with cisplatin alone, cisplatin combined with metformin promoted cell invasion more significantly.

## 4. Discussion

NPC is difficult to detect and diagnose early due to its insidious lesion in the nasopharynx cavity and insignificant early symptoms, and it has a high recurrence risk after initial treatment due to its high metastatic and immune escape potential. With pleiotropic effects, metformin may have beneficial effects on various tissues, but has nothing to do with glucose control [14]. One study has found that metformin can improve cancer outcomes and reduce cancer incidence [15]. Because of its widespread application, metformin has been evaluated in terms of its effects on other diseases. In this study, we analyzed the effects of metformin alone and metformin combined with cisplatin on NPC cells, finding that metformin alone inhibited the activity of NPC cells, and the cell activity decreased with the increase of drug concentration and time. One study has revealed that metformin has anticancer properties, and it exhibits antiproliferative activity by inhibiting intracellular pathways according to in vitro and in vivo experiments [16], and one other study has pointed out that metformin is associated with a reduction in cancer mortality and the effect is dose-dependent [17], which suggested that metformin can inhibit the activity of cancer cells in concentration-dependent and time-dependent manners. It has been verified that metformin can inhibit cell proliferation and induce cell apoptosis by activating the AMP-activated protein kinase pathway [18]. Our results have shown that compared with cisplatin alone, cisplatin combined with metformin could inhibit the proliferation of NPC cells more significantly. One study has found that metformin combined with cisplatin and radiation can further reduce cell proliferation by about 55-60%, significantly stronger than that of each drug alone [19], and one other study has uncovered that metformin combined with cisplatin can not only significantly inhibit cell activity but also induce cell apoptosis [20], which all imply that metformin combined with cisplatin has a strong effect on the biological mechanism of cancer cells. One laboratory study has revealed that metformin inhibits the proliferation of cancer cells and induces their apoptosis [21], and other studies have also concluded that metformin has direct antitumor effect and may inhibit tumor proliferation and induce apoptosis of tumor cells [22, 23].

Therefore, we also evaluated the effects of metformin alone and metformin combined with cisplatin on the migration and invasion of NPC cells, finding that metformin alone inhibited the migration and invasion of cells. One study has also pointed out that in addition to affecting cell proliferation and apoptosis, metformin can also inhibit many other cancer pathways, including blocking the invasion of tumor cells by inhibiting the activation of matrix metalloproteinase 9 [24], which supports that metformin can inhibit cell migration and invasion. One study has revealed that cisplatin combined with metformin can reduce cell activity and metastasis more significantly than cisplatin alone [25]. All these indicate that cisplatin combined with metformin can not only reduce the activity of NPC cells but also inhibit the migration and invasion of them.

Moreover, our apoptosis test results showed that metformin alone induced cell apoptosis. Furthermore, our study also revealed that metformin combined with cisplatin strongly and effectively inhibited cell migration and invasion, which was more significant than that of cisplatin or metformin alone. All the above imply that metformin can promote cell apoptosis. In our study, compared with cisplatin alone, metformin combined with cisplatin was more effective in inducing cell apoptosis, and in other studies, metformin not only weakens the drug resistance of cancer cells to cisplatin but also promotes cisplatin-induced apoptosis [26, 27], which indicate that metformin combined with cisplatin can not only inhibit cell activity, migration, and invasion but also promote cell apoptosis.

## 5. Conclusion

There are still some deficiencies in our study. For example, we have not yet conducted in vivo experiments on the combination of metformin and cisplatin to analyze its therapeutic effects, nor have we studied the specific mechanism of the biological effects of metformin combined with cisplatin on NPC cells. We will continue to carry out research to address the above problems and update our results.

To sum up, cisplatin combined with metformin can inhibit the activity, migration, and invasion of NPC cells and induce their apoptosis.

## Figures and Tables

**Figure 1:** Selection of appropriate cisplatin concentration.

**Figure 2:** Metformin alone inhibited activity of CNE1 cells. Note: ∗ indicates *p* < 0.01*vs.* 0.01 mM metformin; ∗∗ indicates *p* < 0.001*vs.* 0.01 mM metformin.

**Figure 3:** Cisplatin combined with metformin inhibited activity of CNE1 cells. Note: ∗ indicates *p* < 0.01*vs.* cisplatin; ∗∗ indicates *p* < 0.001*vs.* cisplatin.

**Figure 4:** Metformin alone inhibited migration of CNE1 cells. Note: a indicates *p* < 0.05*vs.* the control; b indicates *p* < 0.05*vs.* 0.5 mM metformin; c indicates *p* < 0.05*vs.* 1 mM metformin.

**Figure 5:** Cisplatin combined with metformin inhibited migration of CNE1 cells. Note: a indicates *p* < 0.05*vs.* the control group; b indicates *p* < 0.05*vs.* cisplatin; c indicates *p* < 0.05*vs.* cisplatin+0.5 mM metformin; d indicates *p* < 0.05*vs*. cisplatin+1 mM metformin.

**Figure 6:** Metformin alone inhibited invasion of CNE1 cells. Note: a indicates *p* < 0.05*vs.* the control; b indicates *p* < 0.05*vs.* 0.5 mM metformin; c indicates *p* < 0.05*vs*. 1 mM metformin.

**Figure 7:** Cisplatin combined with metformin inhibited invasion of CNE1 cells. Note: a indicates *p* < 0.05*vs.* the control; b indicates *p* < 0.05*vs.* cisplatin; c indicates *p* < 0.05*vs.* cisplatin+0.5 mM metformin; d indicates *p* < 0.05*vs.* cisplatin+1 mM metformin.

**Figure 8:** Metformin alone induced apoptosis of CNE1 cells. Note: a indicates *p* < 0.05*vs.* the control group; b indicates *p* < 0.05*vs.* 0.5 mM metformin; c indicates *p* < 0.05*vs.* 1 mM metformin.

**Figure 9:** Cisplatin combined with metformin induced apoptosis of CNE1 cells. Note: a indicates *p* < 0.05*vs.* the control group; b indicates *p* < 0.05*vs.* cisplatin; c indicates *p* < 0.05*vs.* cisplatin+0.5 mM metformin; d indicates *p* < 0.05*vs.* cisplatin+1 mM metformin.

## Data Availability

The datasets used and/or analyzed during the current study are available from the corresponding author on reasonable request.
